# Association between TSH-Receptor Autoimmunity, Hyperthyroidism, Goitre, and Orbitopathy in 208 Patients Included in the Remission Induction and Sustenance in Graves' Disease Study

**DOI:** 10.1155/2014/165487

**Published:** 2014-02-18

**Authors:** Peter Laurberg, Birte Nygaard, Stig Andersen, Allan Carlé, Jesper Karmisholt, Anne Krejbjerg, Inge Bülow Pedersen, Stine Linding Andersen

**Affiliations:** ^1^Department of Endocrinology, Aalborg University Hospital, 9000 Aalborg, Denmark; ^2^Department of Clinical Medicine, Aalborg University, 9100 Aalborg, Denmark; ^3^Department of Endocrinology and Internal Medicine, Herlev Hospital, 2730 Copenhagen, Denmark; ^4^Department of Geriatric Medicine, Aalborg University Hospital, 9000 Aalborg, Denmark

## Abstract

*Background*. Graves' disease may have a number of clinical manifestations with varying degrees of activity that may not always run in parallel. *Objectives*. To study associations between serum levels of TSH-receptor autoantibodies and the three main manifestations of Graves' disease (hyperthyroidism, goiter, and presence of orbitopathy) at the time of diagnosis of hyperthyroidism. *Methods*. We describe a cohort of 208 patients with newly diagnosed Graves' hyperthyroidism. Patients were enrolled in a multiphase study of antithyroid drug therapy of Graves' hyperthyroidism, entitled “Remission Induction and Sustenance in Graves' Disease (RISG).” Patients were systematically tested for degree of biochemical hyperthyroidism, enlarged thyroid volume by ultrasonography, and the presence of orbitopathy. *Results*. Positive correlations were found between the levels of TSH-receptor autoantibodies in serum and the three manifestations of Graves' disease: severeness of hyperthyroidism, presence of enlarged thyroid, and presence of orbitopathy, as well as between the different types of manifestations. Only around half of patients had enlarged thyroid gland at the time of diagnosis of hyperthyroidism, whereas 25–30% had orbitopathy. *Conclusions*. A positive but rather weak correlation was found between TSH-receptor antibodies in serum and the major clinical manifestation of Graves' disease. Only half of the patients had an enlarged thyroid gland at the time of diagnosis.

## 1. Introduction

Graves' disease (GD) is a common autoimmune disorder that may affect a number of organs (thyroid, orbit, skin, fingers, and toes) and tissues (e.g., both fat and muscle cells in the orbit). In each location the disease may express a number of clinical manifestations (e.g., in the thyroid: goitre, excessive blood flow, excess thyroid hormone production, and secretion). The disease was originally described as a syndrome consisting of hyperthyroidism, goitre, and orbitopathy [1]. It is now clear that the central element is autoimmunity directed against the TSH-receptor [2], and the vast majority of patients newly diagnosed with Graves' disease have detectable TSH-receptor autoantibodies (TRAb) in serum [3, 4].

The most common manifestation of GD is hyperthyroidism caused by TRAb binding to and activating the TSH-receptor on the follicular cells of the thyroid. Antithyroid drug (ATD) therapy of Graves' hyperthyroidism is in many patients followed by a remission of the autoimmunity of GD with a gradual disappearance of TRAb from the circulation [5]. The tendency to remission is most likely a consequence of making and keeping patients euthyroid [6]. However, the process of remission proceeds very differently in individual patients. In a minority of patients autoimmune stimulation of the thyroid remains excessive [5], whereas at the other end of the spectrum, some patients with mild disease may enter remission even without ATD therapy [7].

The majority of patients with Graves' hyperthyroidism treated with ATD become stably euthyroid within months. A pertinent question in such patients is how long therapy should continue. Based on a limited number of studies [8] current recommendation is that this should be 12–18 months [9]. After withdrawal of ATD, around half of patients will experience a relapse of their hyperthyroidism [8, 9]. Relapse rate of hyperthyroidism after withdrawal of ATD is much higher in some subgroups, such as, for example, patients with moderate to severe Graves' orbitopathy [10]. As a consequence of this some clinics use prolonged ATD therapy in these patients [11, 12]. Clearly, the tools to individualize the duration of ATD therapy in patients with GD need to be improved.

“Remission Induction and Sustenance in Graves' Disease (RISG)” is a multiphase study aimed to improve the knowledge on how GD enters remission in individual patients during ATD therapy and to evaluate if remission can be sustained in a subgroup of patients by a more prolonged low dose ATD therapy.

The present report briefly describes the RISG study and the characteristics of 208 patients with newly diagnosed Graves' hyperthyroidism included in the first phase of the study, RISG1. In this group of patients with newly diagnosed Graves' hyperthyroidism who had been systematically investigated, we studied the association between the three major manifestations of Graves' disease (hyperthyroidism, goitre, and orbitopathy) and the level of TRAb in serum.

## 2. Patients and Methods

### 2.1. Participating Centres

RISG was originally planned to be a multicentre study taking place in several countries. However, because funding to ensure the quality of data was limited, it was decided to restrict the study to the two first clinical centres, Departments of Endocrinology at Aalborg University Hospital and at Herlev Hospital, Copenhagen, both situated in Denmark. Centres were similar in that they both were the primary referral centre for patients with thyroid disease, including Graves' disease for a surrounding population of 250.000–300.000 inhabitants. In Aalborg, general practitioners were informed about the study and a special system was set up to allow immediate referral of patients with newly diagnosed hyperthyroidism to further diagnosis and therapy, thus bypassing normal waiting list. In Copenhagen with no waiting list for such patients, referral followed standard routine; newly referred patients were randomly assigned to a number of specialists in endocrinology, and one of these (BN) included patients in the study.

### 2.2. Inclusion of Patients

Patients were asked to participate in the study when hyperthyroidism had been verified and subtyped as Graves' disease. Subtyping was based on measurement of TRAb in serum (TRAb+ patients were classified as Graves' disease), and no other cause for the hyperthyroidism was identified. RISG1 was in principle a standardized program of ATD therapy which is the routine choice therapy of Graves' hyperthyroidism in Denmark, and all patients accepted to follow the RISG1 program. Exclusion criteria were: age < 18 years, pregnancy within one year, moderate to severe orbitopathy with a need of medical immunosuppressive therapy, intake of drugs affecting the immune system, imminent or manifest thyrotoxic crisis, other severe disease making it unlikely for the patient to be able to follow protocol, thyroid nodules with a need of surgery, intolerance to both Methimazole (MMI) and Propylthiouracile (PTU), previous surgical or radioiodine therapy or ATD therapy for Graves' disease within two years, patient preference of other type of therapy, patient considered unsuited for this type of therapy by responsible MD, TRAb not measurable at time of diagnosis.

### 2.3. RISG Program

The program is illustrated in Figure 1. Patients enrolled in RISG1 were to be treated with partial thyroid block ATD therapy to become euthyroid. In partial thyroid block ATD therapy the dose of ATD is adjusted to allow thyroid hormone production to take place within physiological needs, thereby making and keeping the patient euthyroid. Remission was defined as negative TRAb with a normal TSH on a maximal MMI/PTU dose of 5/100 mg per day. After remission of disease for two months, and when ATD had been given for at least six months, or after a 24 month period of ATD if remission had not occurred, patients would be randomized to either stop ATD or to continue low dose ATD + Levothyroxine, as previously reported [12], for another two years (RISG2). RISG3 was a follow-up of patients without ATD therapy. In case of relapse of hyperthyroidism, patients would be invited to start all over (RISG4) similar to RISG1, followed by RISG5 which is similar to RISG2 (Figure 1).

### 2.4. Investigation at Inclusion in RISG1

Standard history and clinical examination was performed after referral with a focus on verifying hyperthyroidism and diagnosing Graves' disease. A brief questionnaire on previous thyroid disease, intake of medication, including estrogen and nutritional supplements, smoking habits, other diseases, and family history of thyroid disease was filled out. Thyroid ultrasonography was performed with the measurement of thyroid volume [13] and the eyes were evaluated for signs and symptoms of Graves' orbitopathy. New blood samples were taken for measurement of serum T4, T3, TBG or T3-test, TSH, TRAb, TPO antibodies, liver function tests, haematological parameters and ANCA. TRAb was measured using a receptor assay (DYNOtest TRAK, Thermo Fisher, Berlin, Germany) (TRAb ≥ 1.0 IU/L being considered TRAb positive) [3], TPO-Ab (detection limit 30 kU/L [14]) by KRYPTOR antibody tests (Thermo Fisher, Berlin, Germany). Serum T4 concentration (reference range: Aalborg 60–140 nmol/L, Copenhagen 60–140 nmol/L), T3 (reference range: Aalborg 1.1–2.5 nmol/L, Copenhagen 1.0–2.6 nmol/L), and TSH (reference range: Aalborg 0.30–4.5 mU/L, Copenhagen 0.40–4.0 mU/L) were measured by standard high capacity tests (Aalborg, Roche Diagnostics Elecsys; Copenhagen, Immulite 2500, chemiluminescent enzyme immunoassay).

Clinical routine in most hospitals in Denmark is to use total T4 and T3 for diagnosis and treatment of thyroid disease with a single measurement of TBG or a T3 test to evaluate thyroid hormone binding capacity. In the present study, 32 women used estrogen containing medication and they had high serum TBG. Apart from this, binding of thyroid hormones in serum was normal. In the data analyses including serum T4 and T3, participants who took estrogens were excluded leaving 176 for analyses. Serum T4 and T3 values used in the present study were the last set of test results obtained before initiation of therapy.

### 2.5. Statistical Analysis

Data were analyzed using IBM SPSS statistics versus 21.0. Nonparametric tests were used for comparisons and correlation analyses. The study was approved by the North Denmark Region Committee on Health Research Ethics (VN-20060062) and registered in ClinTrial.gov (NCT00796913).

## 3. Results

During the period January 11, 2007 to June 6, 2011, 208 patients with newly diagnosed hyperthyroidism caused by Graves' disease were included at the centres in Aalborg and in Copenhagen. Characteristics of the patients are given in Table 1. Eighty percent of participants were included in Aalborg, with no difference in most of patient characteristics between centres. Patients from Copenhagen were slightly less hyperthyroid and had a lower thyroid volume and a lower frequency of eye changes. In addition, they had a lower body weight and BMI.

### 3.1. Thyroid Volume

The distribution of thyroid volume in patients at entry is depicted in Figure 2. Using cut-offs developed to depict thyroid enlargement, this was found in 46.9% of men (volume > 25 mL [15]) and 53.4% of women (>18 mL [15]). Thyroid volume was larger in male (median thyroid volume 24.5 mL (range 9.9–105)) than in female (19.2 (5.6–112)) patients (*P* = 0.013).

Thyroid volume correlated positively with body weight in women (Spearman correlation (*r*_*s*_) = 0.15, *P* = 0.049), but this did not reach statistical significance in men (*r*_*s*_ = 0.21, *P* = 0.25), with TRAb (see below), with serum T4 and T3 (see below), with TPO-Ab (*r*_*s*_ = 0.24, *P* = 0.001), and with the presence of eye changes (*r*_*s*_ = 0.17, *P* = 0.017).

### 3.2. TSH-Receptor Antibodies

The distribution of TRAb values is shown in Figure 3. TRAb values correlated positively with serum T3 (*r*_*s*_ = 0.54, *P* < 0.001) and serum T4 (*r*_*s*_ = 0.31, *P* < 0.001), with the presence of eye signs and symptoms of orbitopathy (*r* = 0.15, *P* = 0.036), and with thyroid volume (*r* = 0.25, *P* < 0.001). No correlation was observed with age, sex, body weight, smoking, previous ATD therapy, family occurrence of Graves' disease, or serum TPO-Ab (*r* = 0.13, *P* = 0.06).

### 3.3. Serum T4 and T3

Serum T3 was in general more elevated than serum T4 with 57% of T3 values being more than twice the upper normal limit. This was only 16% of serum T4 values. Both serum T4 and T3 correlated positively with TRAb (see above) and with thyroid volume (T4: *r*_*s*_ = 0.49, *P* < 0.001; T3: *r*_*s*_ = 0.48, *P* < 0.001). Serum T3 correlated negatively with age (*r*_*s*_ = −0.21, *P* = 0.005), whereas no correlation was observed between serum T4 and age (*r*_*s*_ = −0.06, *P* = 0.43). A high internal correlation between T3 and T4 was present (*r*_*s*_ = 0.76, *P* < 0.001). No correlation was found with TPO-Ab or any of the other variables investigated. The ratio T3/T4 in serum correlated to the severity of disease as evaluated by the three main disease manifestations. (T4: *r*_*s*_ = 0.20, *P* = 0.007; thyroid volume: *r*_*s*_ = 0.32, *P* < 0.001; orbitopathy present: *r*_*s*_ = 0.15, *P* = 0.041).

## 4. Discussion

We describe the characteristics of a group of patients with newly diagnosed hyperthyroidism caused by Graves' disease. The patients were prospectively and systematically investigated as part of inclusion in a two-centre multiphase study that aimed to improve the tailoring of ATD therapy to individual patients.

### 4.1. The “Merseburg Triade”

A consistent part of early description of patients with Graves' disease was the presence of symptoms and signs of hyperthyroidism, eye changes corresponding to Graves' orbitopathy, and diffuse goitre. This combination was brought forward by Parry [16], by Basedow [17], and by Graves [18]. Named after the German city where Basedow practised medicine, the combination of disease manifestations has been called the Merseburg triade [19].

The patients in the present study were recruited based on being hyperthyroid, and this is undoubtedly the most common manifestation of Graves' disease. In our epidemiological study of patients with moderate end severe Graves' orbitopathy 87% of patients suffered from hyperthyroidism, whereas 6% were hypothyroid (presumably caused by TSH-receptor blocking antibodies or thyroid autoimmune destruction) and 7% euthyroid [20]. In population studies it is uncommon to find TRAb positivity even in patients with goitre [21], but around 10% of patients with newly diagnosed hypothyroidism are TRAb positive [3].

Thus, hyperthyroidism is the most common manifestation of Graves' disease (defined as an autoimmune disease caused by TSH-receptor autoimmunity) being present in around 90% of patients, whereas hypothyroidism develops in 5–10% of patients. Notably, a few percent of patients treated for a period with ATD for hyperthyroidism caused by Graves' disease may develop hypothyroidism during the course of ATD [22].

Goitre is also a classical, although less consistent manifestation of Graves' disease. In the present study only around half of the patients had an enlarged thyroid when measured by ultrasonography. Still, the thyroid may have been larger than before disease developed, but we have no data on this. Previous studies have also described that a fraction of patients may not have goitre at the time of diagnosis of Graves' hyperthyroidism [23, 24].

The third of the major manifestations, orbitopathy, was observed in 25–30% of RISG patients at the time of diagnosis. All had mild orbitopathy. We did not include patients with moderate and severe orbitopathy in the RISG study, because such patients would be treated with immune modulating drugs that might alter the course of the disease. The occurrence of the more severe forms of Graves' disease is rather low, and orbitopathy is often not present in severe form at the time of diagnosis of hyperthyroidism [20].

### 4.2. Correlation with TRAb

Our study of correlation between the various degrees of manifestations and the level of TRAb at diagnosis corroborated the central role of TSH-receptor autoimmunity in Graves' disease. A clear positive correlation was observed between the concentration of TRAb in serum and first, thyroid volume, second, degree of biochemical hyperthyroidism, and third, the presence of eye signs. However, although statistically significant some of the correlation coefficients were rather low. Thus, factors other than the level of TRAb were also of major importance for the clinical expression of disease.

Serum T3 correlated negatively with age. This may be due to a higher prevalence of concomitant diseases in the elderly participants [25]. Serum T3 was more elevated in the hyperthyroid patients than serum T4 which is in agreement with previous findings [26] including those of a population based study [27]. The pattern is presumably caused by high deiodinase type 1 activity in the hyperactive thyroid that deiodinate T4 to T3, that is, both T4 released from thyroglobulin during secretion and T4 taken up by the hyperactive thyroid from circulation [28]. Corresponding to this, the T3/T4 ratio in serum was to some degree a measure of disease activity with a positive correlation to thyroid volume, TRAb, the presence of orbitopathy, and serum T4.

### 4.3. Study Limitations

The patients included in the present study were referred to hospital by general practitioners, and some degree of referral bias may be present. Graves' disease patients referred to hospital may be younger and more severely hyperthyroid than the average patient [29]. The small difference in characteristics between patients included in Aalborg and in Copenhagen may suggest that some degree of patient selection indeed took place. We included only patients who had measurable TRAb in serum. In the order of 5% of patients with newly diagnosed Graves' hyperthyroidism are TRAb negative using the TRAb assay employed in the present study [3]. Overall, these tend to be patients with mild disease [30]. A subgroup of patients took estrogens which increases serum TBG and total thyroid hormone concentration. We excluded these patients in the analysis of T4 and T3 correlation. We correlated the T3/T4 ratio in serum to serum T4 even if random variation in serum T4 may give a significant covariation. However, such covariation will tend to give a negative correlation, whereas we observed a positive correlation. The present study gave no information on the mechanism behind the correlation between TRAb and the various manifestations of Graves' disease. Whereas this is logical when it comes to the state of hyperthyroidism and the size of the goitre, the mechanisms leading to orbitopathy and the other more rare manifestations are less clear.

## 5. Conclusion

We describe a large cohort of patients with newly diagnosed Graves' disease who entered a study aimed to improve quality of ATD therapy. Analysis of patient characteristics corroborated the central role of TSH receptor autoimmunity in Graves' disease and the association between the three common manifestations of Graves' disease. Future results of the RISG study may clarify if TRAb levels and the various clinical manifestations at entry are useful for tailoring duration of ATD therapy to individual patients with hyperthyroidism caused by Graves' disease.

## Figures and Tables

**Figure 1:** Overview of the RISG study. The present study describes the 208 patients included.

**Figure 2:** Distribution of thyroid volumes (5 mL intervals) in patients with newly diagnosed hyperthyroidism caused by Graves' disease and enrolled in the RISG study. Male patients: dark grey, female patients: light grey. Among the men, 46.9% had enlarged thyroid (>25 mL), whereas this was 53.4% in the women (>18 mL).

**Figure 3:** Distribution of serum TRAb values in patients with newly diagnosed hyperthyroidism caused by Graves' disease and enrolled in the RISG study. According to inclusion criteria, none had TRAb < 1.0 IU/L. Up to 40 IU/L, intervals are 2.5 IU/L wide. At 40 IU/L and above, intervals are 20 IU/L wide.

**Table 1:** Characteristics of patients included in RISG1.

	Aalborg	Copenhagen	All	*P*
Participants, *n* (%)	167 (80.3)	41 (19.7)	208 (100)	—
Sex, F/M (% F)	138/29 (82.6)	38/3 (92.7)	176/32 (84.6)	0.15
Age years, median (IQR)	44 (34–53)	47 (36–55)	45 (35–53)	0.55
Previously hyperthyroid, *n* (%)	12 (7.2)**	0 (0)	12 (5.8)	—
Smoker, *n* (%)	45 (26.9)	11 (26.8)	56 (26.9)	1.00
Estrogen use, *n* (%)	29 (21.0)	3 (7.9)	32 (18.2)	0.93
GD in 1st generation relatives, *n* (%)	42 (25.3)*	11 (26.8)	53 (25.5)	0.87
Body height cm, median (IQR)	168 (163–173)	167 (162–172)	168 (163–172)	0.25
Body weight kg, median (IQR)	65.3 (57.8–78.1)	60.0 (53.5–68.5)	64.5 (57.5–75.9)	0.007
BMI kg/m^2^, median (IQR)	23.5 (21.1–26.2)	22.0 (19.9–23.8)	22.9 (20.8–26.0)	0.011
Graves' orbitopathy, *n* (%)	51 (30.5)	5 (12.2)	56 (26.9)	0.018
S-T4 nmol/L, median (IQR)	213 (177–269)	189 (167–238)	201 (175–255)	0.086
S-T3 nmol/L, median (IQR)	5.5 (4.3–7.5)	5.0 (3.5–6.3)	5.4 (4.2–7.1)	0.021
S-TRAb IU/L, median (IQR)	9.1 (5.1–14)	9.7 (5.4–22)*	9.1 (5.2–15.2)	0.37
S-TPO kU/L, median (IQR)	277 (33–2295)	230 (30–3600)***	266 (30–2717)	0.80
Thyroid volume mL, median (IQR)	21.1 (15.8–34.3)*	16.0 (10.0–24.0)*	20.0 (14.5–31.9)	<0.001

*P* for comparison between Aalborg and Copenhagen participants using Mann-Whitney *U* test or the Pearson *χ* ^2^/Fisher's exact test as appropriate. F: female. M: male. IQR: 25–75% interval. GD: Graves' disease.

*One value missing.

**Two values missing.

***Three values missing.
